# Analysis of Emotional Stress of Teachers in Japanese Teaching Process Based on EEG Signal Analysis

**DOI:** 10.1155/2022/2593338

**Published:** 2022-06-29

**Authors:** Jie Dong

**Affiliations:** School of Foreign Languages Studies, Wenzhou Medical University, Wenzhou, Zhejiang 325035, China

## Abstract

The construction direction of Japanese teaching evaluation system based on hybrid teaching mode is to give full feedback to teaching process, diversify evaluation subjects and evaluation methods, and obtain comprehensive and objective evaluation results. Compared with most similar studies, more EEG data of teachers' emotional stress relief and healthy people in Japanese teaching process were collected, and a large number of features were extracted. An experiment of teachers' emotional stress relief recognition in Japanese teaching process based on EEG signal was designed. The feature selection algorithm was used to screen the EEG feature combinations of teachers' emotional stress relief and healthy subjects, and the classification experiment was carried out to verify the difference. Finally, this paper uses the feature selection algorithm of tree model and the random forest model classifier to establish the recognition model of teachers' emotional stress discharge in Japanese teaching process based on EEG signals and achieves the effect of more accurate recognition of teachers' emotional stress discharge in Japanese teaching process. First, the connotation, value, and influencing factors of teachers' emotion management ability are logically integrated and systematically expounded. Second, based on emotional psychology, emotional intelligence theory, psychotherapy theory, and management theory, teachers' emotional management ability is constructed according to the three-dimensional structure theory of intelligence and information processing theory. It is constructed from three dimensions: object dimension (teachers themselves, students, and students), content dimension (positive and negative emotions), and operational dimension (emotional perception, emotional understanding, emotional expression, and emotional regulation).

## 1. Introduction

With the development and progress of society, the role of talents has become prominent, and the country and society have paid unprecedented attention to education, which has brought various pressures and challenges to the profession of teachers. Especially in recent years, with the in-depth development of new curriculum reform, teachers have to face various reforms while completing their teaching tasks. Excessive work pressure increases the frequency of teachers' emotional fluctuations. However, Japanese teachers are burdened with complex and heavy educational tasks, such as high work intensity, complex work process, long periodicity, and lack of timely recognition of achievements. At the same time, the teachers of Japanese language teaching are also facing strong pressure of entering school, and various pressure situations make teachers' emotional problems increasingly accumulate and highlight. As one of the social members, teachers play multiple roles in social life, the role and the role of conflict and contradiction between and interpersonal complicated social life, which makes teachers produce many contradictions in the work and life and cause a series of emotional responses and wave and eventually to cause a lot of emotional problems. As the ability to process and deal with emotional information, the research on teachers' emotional management ability is helpful to adjust and alleviate teachers' emotional problems.

Teachers' emotional stress in the process of Japanese teaching is closely related to brain activity [1, 2]. Numerous studies have shown that brain circuits control the production of emotional behavior. Therefore, through the study of EEG signals, teachers' emotional stress tendency in Japanese teaching can be objectively and effectively identified. To pick up the relevant electrical signals, researchers use a variety of techniques to induce mood changes. At present, there are many ways to induce emotions. Sixteen subjects were subjected to picture stimulation to study the difference of EEG signals of different facial expressions under picture stimulation [3]. Using the method of auditory stimulation, the change of Alpha band power of EEG in college students was studied [4]. An emotion induction experiment was designed to explore the EEG synchronization between different brain regions when different emotions were perceived. Although visual stimulation, auditory stimulation, and combination of audio-visual and visual stimuli can all make subjects produce changes in EEG signals, visual and picture stimulation can better induce relevant emotions of subjects [5]. At the same time, studies have shown that there are differences in the autonomic nervous system between positive and negative emotions induced by pictures [6]. For Japanese teaching process of teachers' emotional stress research also has a lot of progress, the study of Japanese teaching process of teachers' emotional stress disorder found that under the Gamma spectrum, Japanese teaching process teachers' emotional stress disorder with different hemisphere advantage, namely, in the negative emotional pictures, the left hemisphere is more active, and in positive mood pictures, the activity intensity of the right hemisphere was more significant [7]. Although there are many related researches on teachers' emotional stress disorder in the process of Japanese teaching, the current research on teachers' emotional stress in the process of Japanese teaching rarely focuses on male and female college students. Few studies have been conducted to define the temporal relationship between teachers' emotional stress and emotional tendencies in the Japanese teaching process. Therefore, in this study, picture stimulation is used to induce EEG signals, and male and female college students are taken as experimental objects to conduct time-frequency analysis of their EEG signals in frequency band. This paper tries to find the emotional features with feasible high recognition rate for predicting teachers' emotional stress in Japanese teaching process (teachers' emotional stress tendency in Japanese teaching process) at certain time periods with significant correlation in Theta, Alpha, and Beta bands.

Hybrid teaching mode is formed under the support of information technology, which changes the disadvantages of traditional teaching “time and space limitation” and can obtain higher teaching efficiency under flexible and changeable arrangement. The construction of Japanese teaching evaluation system based on hybrid teaching mode should not only conform to the characteristics of the mode but also fully evaluate the operation of the mode. Only in this way can the hybrid teaching mode play a greater role in Japanese teaching. From the current situation, many universities have set up Japanese major, so the research on Japanese teaching evaluation system has broad application space and can provide strong support for the better development of Japanese teaching. In order to diagnose the emotional stress of teachers in Japanese teaching more conveniently and to simplify the EEG collection process, it is of great significance to study an EEG recognition model with fewer channels. Therefore, we confirm the title of this paper: research and realization of emotional stress disorder recognition of teachers in Japanese teaching process based on EEG signals, aiming to provide an objective and convenient way to assist doctors in diagnosing emotional stress disorder of teachers in Japanese teaching process. In addition, the model channel studied in this paper is also a reference for the EEG channel concerned by simplified portable EEG devices.

## 2. Related Work

With the deepening of the research, the related emotion management research is also gradually developed. Foreign scholars' definition of emotion management can be divided into three categories. The first type is service management, which emphasizes that emotional management is an activity conducive to one's own survival and development and serves individuals [8]. Individuals manage their emotions according to the relationship between social situation and themselves and their own coping ability. The second type is trait management, which emphasizes certain features or features of emotion management. Emotional management is a subordinate concept of emotional intelligence and one of the components of emotional intelligence. From the perspective of the dynamic characteristics of emotional management, it is considered that emotional management is a dynamic organizational system occurring inside and outside consciousness, including physiological, cognitive, experiential, and behavioral reactions [9]. The third is adaptive management, which emphasizes that emotional management is a process of adapting to social reality. Emotion management is to flexibly respond to positive or negative emotions in a socially acceptable way according to needs [10]. Emotion management is an activity process that adapts to social reality. It requires people's emotional response to be flexible, adaptive, and appropriate, so that people can adapt to changing social situation quickly and effectively in an organized and constructive way.

In the hybrid teaching mode, students can not only further expand their learning space but also obtain sufficient learning resources relying on Internet channels. However, it should be noted that teachers' emotions in the process of Japanese teaching based on EEG analysis have both advantages and disadvantages, because while students enjoy online “welfare,” they also need to face the impact of online complex information, especially those bad information will bury hidden dangers to students' physical and mental health [11]. Under such circumstances, the Japanese teaching evaluation system based on the hybrid teaching mode needs to be able to control the teachers' emotions in the process of Japanese teaching under the analysis of EEG signals, make a comprehensive and objective evaluation of students' online learning process, and help teachers make targeted responses [12]. In order to achieve this goal, conventional offline evaluation methods are not applicable. Only by developing evaluation methods based on online characteristics that are suitable for the analysis of EEG signals in the process of Japanese teaching can they play a corresponding role. For example, the current MOOC and SPOC teaching data statistics platforms are commonly used evaluation methods [13]. These methods can not only evaluate students' performance in all aspects based on online data but also provide students with teaching content that can stimulate students' interest and enthusiasm based on their needs, so that students can get better training [14]. Hybrid teaching mode is a combination of online and offline teaching, therefore in the construction of teaching evaluation system, cannot simply “an almost,” but is based on the specific characteristics of the adopted corresponding evaluation concept and evaluation methods, such as offline teaching teachers will real contact with the student, the teacher to the student “move” to; however, in the process of Japanese teaching teachers' emotions based on EEG analysis, teachers can only rely on relevant virtual data to understand students' process performance [15]. Although the evaluation methods are different, the evaluation objectives are the same, that is, to optimize students' learning effect, improve teaching quality, and so on. Specifically, the principle of consistency of objectives mainly requires that online and offline teaching evaluation methods do not have conflicts and truly “work together” [16]. For example, offline exams are easy to be controlled, and students will abide by the examination rules and regulations under the strict supervision of teachers. However, online exams are “controlled remotely,” so it is difficult for teachers to manage students properly. In view of this situation, it is necessary to adjust the content of the examination questions. For example, the offline examination questions can take the basic knowledge of language as the main object of investigation, while the online examination questions focus on the investigation of students' oral expression.

In the context of the current hot research on artificial intelligence, machine learning methods have been widely applied, and the field of artificial intelligence-assisted diagnosis and treatment has achieved rapid development. In addition, the emotional stress relief of teachers in the process of Japanese teaching has also been widely concerned in recent years. Many researchers in this context have tried to use machine learning method to detect teachers' emotional stress relief in Japanese teaching process from EEG signals in resting state [17]. Some recent literatures have proved that it is a feasible method to use resting state EEG detection and classifier to identify teachers' emotional stress relief during Japanese teaching. In the resting state EEG samples including 34 cases of teachers' emotional stress relief in the process of Japanese teaching and 30 cases of normal controls, the classification accuracy of 93.33% was achieved by using relative wavelet energy and Alpha frequency power [18, 19]. In addition, nonlinear features such as fractal dimension and maximum Lyapunov index were used in EEG data collected from 15 and 15 normal people, and the recognition accuracy of SVM classifier reached 98% [20]. Among 14 normal people, the highest classification accuracy of 91.4% was obtained by analyzing the relative power spectrum density and coherence of EEG signals [21]. In each study, features were extracted from EEG signals in the resting state to analyze the emotional stress of teachers in the process of Japanese teaching. In most cases, machine learning classifiers are used to calculate some time domain and frequency domain features to classify. It can be seen that more and more Japanese teaching process teachers' emotional stress relief and recognition began to use machine learning. In recent years, the development of deep learning has made great progress, and there are a few literatures that use deep learning methods to directly recognize EEG signals without noise. The neural network combined with convolutional neural network and long and short-term memory neural network was used to conduct research on EEG data sets collected from 15 and 15 healthy people, achieving the highest accuracy of 99.12% [22]. There is also some progress in the research on teachers' emotional stress in the process of mild Japanese teaching. In some literatures, EEG was collected under the condition of stimulation, and deep neural network was used to study teachers' emotional stress in the process of mild Japanese teaching and the normal control group (24 cases of teachers' emotional stress in the process of mild Japanese teaching). In terms of domestic and foreign studies, many literatures have proved that they have extracted appropriate EEG features as biomarkers for teachers' emotional stress relief in the process of Japanese teaching, with high recognition accuracy. However, almost all the studies were conducted on the EEG data set of few healthy teachers and teachers' emotional stress relief in Japanese teaching process, and quite a few studies were conducted on the EEG data of more than ten or twenty healthy teachers and teachers' emotional stress relief in Japanese teaching process [23–25]. This may be related to the difficulty of collecting EEG signals and the sensitivity of volunteers' physiological data. Open source EEG data sets on the Internet are mostly EEG data of healthy people, and few EEG data of teachers' emotional stress relief during Japanese teaching. In addition, there are few studies on the location and number of brain regions and EEG signal channels.

## 3. Electroencephalogram Analysis of Japanese Teaching Process Teacher Emotional Stress Relief Technology Analysis

### 3.1. Analysis of EEG Signal Characteristics

Volunteers were instructed to sit in a quiet room with no sound or signal. We helped the subjects to wear EEG caps and apply conductive paste to the corresponding EEG electrodes until the electrode impedance of all EEG channels met the requirements and EEG was collected. The process of EEG data collection was to use a 10-20 system to record the EEG data of 64 channels of the subjects. The data were first collected when the subjects opened their eyes for 3 minutes and then collected when the subjects closed their eyes for 3 minutes. The whole preparation stage takes about 20 minutes, plus the 6 minutes of actual EEG collection and the time of filling in the scale, each subject participates in the experiment for about 40 minutes. At this time, the subject volunteers left, and we cleaned the EEG cap and renamed the EEG data according to the format, as shown in Figure 1.

Detrended fluctuation analysis (DFA) was used to analyze the long range correlation of time series. One of the advantages of DFA method is that it can filter the trend components of each order in the signal sequence and detect the long range correlation with noise ave and polynomial trend signal superposition y, which is suitable for the long range power law correlation residue analysis of nonstationary time series.

(1) $$\begin{array}{c} X\left(t\right)=\overset{t}{\underset{i=1}{\sum }}\left(y\left(i\right)-\text{ave}\right). \end{array}$$

(2) $$\begin{array}{c} \text{Residue}=\sum \left(x\left(t\right)-X_{k}\left(t\right)\right). \end{array}$$

Then, the window function *W* (*n*) is added to each EEG data segment, and the periodic graph of each segment is obtained. The periodic chart of paragraph I:

(3) $$\begin{array}{c} x_{i}\left(w\right)=\frac{1}{I}\overset{M}{\underset{0}{\sum }}x\left(t\right)w\left(m\right),i=1,2.\cdots M. \end{array}$$

The absolute centroid is the dot product of frequency *F* and power PSD in the frequency band.

(4) $$\begin{array}{c} \text{Centroid}=\frac{\sum_{f2}\text{P}\text{SD}\left(Fi\right)}{\sum_{fh}\text{P}\text{SD}\left(Fh\right)}. \end{array}$$

The first step in the construction of Japanese teaching evaluation system is to divide teaching activities and establish competence objectives based on teaching activities. In offline Japanese teaching, teaching activities include classroom tests, group tasks, self-evaluation and interaction, simulation, summary and reflection, final comprehensive project, and demonstration project. Japanese analyzes teachers' emotions in the teaching process. Teaching activities include reading digital resources, unit operation, homework mutual, unit test, final test, video of primary and secondary tests, classroom test, BBS answering questions, raising questions, and resource analysis. The goal of search and matching ability is “autonomous learning, knowledge, skills, knowledge skills and habit Formation,” “Communication and collaboration,” “knowledge skills and habit formation,” “knowledge skills,” “communication, interaction, analytical thinking,” and “information literacy, analytical thinking”.

### 3.2. Theoretical Model of Teachers' Emotion Management Ability

After the correlation between teaching activities and ability objectives, the key indicators should be determined on the basis of both, and then the corresponding assessment methods should be selected according to the content of the indicators. In this process, the key indicators should not only reflect the teaching situation but also meet the needs of the actual platform, such as online platform. The index content should not only be easy to quantify but also be able to truly measure the relevant situation. For example, the “online duration” index is relatively difficult to quantify. However, if it is unscientific to measure students' learning attitude, attendance rate, and learning efficiency by relying on this index, comprehensive consideration should be carried out in combination with other indicators. In specific view, Japanese teaching evaluation system can be divided into online key, noncritical online, and offline key indicators, offline noncritical indicators, and evaluation methods including formative assessment and summative assessment, such as in online critical index determination, unit testing, unit operation, and the final test are the determination of the content, formative evaluation and summative evaluation are the specific evaluation methods.

The purpose of weight setting is to determine the proportion of assessment indicators in the evaluation system. To get scientific and reasonable evaluation result, need comprehensive consideration when weighting, such as in the online learning evaluation for students, “the online time” weight proportion should be reduced, and the weight of “in-class quiz” proportion should be improved, because “in-class quiz” better reflect the student is listening. In offline teaching, the proportion of the weight of “teacher evaluation” should be reduced, while the proportion of the weight of students' mutual evaluation should be increased, which can not only stimulate the enthusiasm of students to participate in the evaluation but also enhance the objectivity of the evaluation results, so that students can get comprehensive and objective evaluation. The weight setting of assessment indicators is not fixed, but should be flexible based on the specific situation. For example, in Japanese teaching, the evaluation of basic language knowledge should be based on grammar, vocabulary, and other test scores, but in the evaluation of oral expression ability and writing ability, the actual effect on site should be an important indicator.

All 5,518 computational features were obtained. It is necessary to determine which feature subset or channel EEG signals best describe the differences between EMD teachers and healthy controls in Japanese teaching, i.e., a small number of EEG channels are selected by feature selection. Three different feature selection models were tested in order to find a better combination of EEG features and provide the best recognition effect of emotional stress disorder in Japanese language teaching. In addition to feature selection methods in statistics, this paper also tries to use machine learning model to assist feature selection, and Sklearn package also provides corresponding methods.

#### 3.2.1. Linear Feature Selection Based on L1 Regularization

Coefficients of linear models were used to screen for EEG features. The more important the feature, the larger the coefficient in the model. The coefficients for features unrelated to the predicted results are small. A sparse matrix is formed if there are more zeros. However, in most of the actual data, there are multiple interrelated features, so the model will become unstable. A little noise in the data may lead to huge changes in the model, which will make the prediction accuracy of the model very low. Regularization addresses this problem to prevent overfitting and improve generalization.

(5) $$\begin{array}{c} \min\frac{1}{2n_{\text{sample}}}{\left|w\left(n\right)-y\right|}^{2}+\alpha {\left|w\right|}^{2}. \end{array}$$

In combination with the accuracy of classification, the parameters of the three feature selection methods are repeatedly adjusted, and the final feature selection parameters are shown in Table 1.

7 positive pictures and 7 negative pictures were formed into a stimulus sequence, each picture appeared 55 times, and the stimulus sequence appeared 4 times in succession. The pictures were randomly drawn. In order to calm the emotions of the subjects, there was a fuzzy picture between the pictures of different groups, and the time of the picture appeared was 5 s. The stimulus design is shown in Figure 2.

Through interviews with teachers in a school, it is found that most teachers are aware that negative emotions need to be regulated, but they are not aware of the regulation and maintenance of positive emotions. When asked “how to regulate their negative emotions,” the teachers' answers are shown in Table 2.

When asked “how do you regulate the negative emotions of individual students and student groups,” the teacher's answers are shown in Table 3.

Brain electrical signal is a signal of change over time, every moment is composed of different frequency components, so only in the time domain or frequency domain cannot be a comprehensive expression of the “real” on brain electrical signal, and the time-frequency analysis of signal in time and frequency range can be displayed at the same time, namely, the signal in time and frequency domain of the plane. It can be expressed as a function with time and frequency as independent variables to better show the change of signal frequency along the time axis. Moreover, the EEG signals of many lesions are presented in transient form, and time-frequency analysis can be used to discuss and study the signals more intuitively and accurately. In order to study the changes of EEG signal energy of negative images and positive images during Japanese teaching, event-related spectral perturbation was used to analyze EEG signals of related emotions. In this analysis method, the energy spectrum of experimental data is divided into multiple segments, then these segments are superimposed on an average basis, and the change value of the energy spectrum is calculated. If the energy spectrum changes, it indicates that there is a time-locked relationship here. Otherwise, there is no lock-time relationship. The calculation method is as follows:

(6) $$\begin{array}{c} \text{ERSP}=\frac{1}{n}\sum {\left|Y_{k}\left(t,k,c\right)\right|}^{2}. \end{array}$$

The cultivation and improvement of teachers' emotional management ability need a long time of accumulation and cultivation, which not only requires a solid emotional theory as the foundation but also requires repeated practice and revision in teaching. The cultivation of teachers' emotional management ability can be divided into preservice and postservice stages. Preservice training is the initial cultivation stage of teachers' emotional management ability, while postservice training is the development and improvement stage of teachers' emotional management ability. Different emphases make the training contents and teaching methods of each stage show different trends. Preservice training, as the cultivation and preliminary cultivation stage of teachers' emotional management ability, mainly focuses on theoretical learning. On the basis of mastering subject knowledge and professional knowledge, courses related to emotion and emotion are offered to enable preservice teachers to have certain emotional management knowledge, laying theoretical foundation for the cultivation of emotional management ability. In terms of teaching methods, the practice of education should be strengthened while teaching theoretical knowledge. Theoretical part of the teaching to strengthen the teaching model and introducing case teaching, make it to have a comprehensive understanding of theoretical knowledge, at the same time, in the practice through the education practice, a variety of forms such as simulation teaching, the teaching can not only increase contact with teachers and students, make it a better understanding of teachers' emotional impact on teaching and role, and enhance the consciousness of manage their emotions; moreover, it can feel the demonstration of mature teachers' classroom emotion and its regulation and understand the generation and development of teachers' emotion management ability. Postcareer training is the reconstruction of the teacher's emotion management ability and enhance stage, the teacher may go through self training, school-based training, teacher training, peer exchanges, and experts in various training modes to improve their mood and their ability to manage, in the mode of training, pay attention to the communication with teachers and discussed, such as through teaching requires teachers to review what happened in the discussion and evaluation, reflect on your emotions and think of strategies to adjust. Descriptive statistics and analysis are made on the questionnaire survey results of the current situation of teachers' emotion management, as shown in Table 4.

Look from the research data on average, Japanese teaching teachers' emotion management level as the growth of the age and teaching experience will be from high to low to high state of development, 20 to 30 years old of young teachers' emotional management level, the highest in this age group teachers usually is just the “novice” to be going to work, because it has the high work enthusiasm, emotion expression way is more exposed, enthusiasm, extroversion, and liveliness make them emotionally passionate, willing to show and hope for recognition, so that they have a good emotional management level. Key teachers aged 30 to 40 have the lowest emotional management level. With the increase of age and experience, Japanese teachers are under increasing pressure from all sides, and the factors affecting emotional management are increasing and strengthening. Middle-aged and elderly teachers aged 40-50 are more stable in their emotions, more reserved in their emotional expressions, and further reduce the frequency of interaction with students. Their emotional control methods and abilities are also more rich and mature. Teachers should pay attention to guide and organize classroom teaching activities that students participate in, correct mistakes in time, and give evaluation according to students' performance. Evaluation is the affirmation and encouragement of students' participation in classroom activities. The classroom teaching process is shown in Figure 3.

The whole process of classroom teaching is guided by teachers, emphasizing the dominant position of students in learning and creating a Japanese learning environment through the assistance of network resources. The application of network resources in classroom teaching can successfully complete the teaching tasks, achieve the teaching objectives of this class, improve the quality of classroom teaching, and achieve teaching effects.

## 4. Example Verification

In order to make the experimental results more clear, ERSP (event-related spectral power) results were statistically analyzed. The statistical analysis method used in this experiment is *T*-test. *T*-test is a parameter test, which deduces the probability of the occurrence of difference according to the *T*-distribution theory, so as to compare whether the difference between two means is statistically significant. The P-P method draws a graph based on the relationship between the cumulative ratio of a variable and the cumulative ratio of a given distribution. The p-p diagram is used to verify that the data conforms to the specified distribution. Since normal distribution test is the premise and basis of *T*-test analysis, P-P method of normal probability graph is used to test the normality of the average power spectral density value obtained in SPSS19.0, and the results are shown in Figure 4. Since the scattered points are clustered around the fixed line, the data can be considered as approximately normal distribution. *P* < 0.05 indicates significant correlation, and *P* < 0.01 indicates extremely significant correlation. Figures 5 and 6 show ERSP results after *t* test at F3 poles. When a red dot appears in the results of statistical analysis, it represents a significant correlation.

The subjects were divided into the experimental group and the normal group (14 subjects in the normal group and 5 subjects in the experimental group with the tendency of emotional stress relief in Japanese teaching process under the analysis of EEG) and analyzed statistically. After statistical analysis, it can be seen (Table 5) that there is no statistical significance in occipital lobe, but there is statistical significance in other brain regions (*P* < 0.05), and there is highly statistical significance in AF3, F7, F3, FCS, T7, P7, and AF4 (mostly left brain) when viewing positive images (*P* < 0.01). However, the pictures of teachers' tendency to deal with emotional stress in the process of Japanese teaching with EEG analysis were particularly significant at F3, FCS, and F8. At the same time, it is found that there is almost no statistical significance in the Theta band during the event-related spectrum disturbance analysis.

ROC curves on the test set and all data sets are shown in Figure 7. The curve on the upper left is the ROC curve of the model on all data sets containing the training set of the test set, and the other is the ROC curve on the test set. As you can see from the graph, the curve near the upper left is made up of larger AUG, which is more accurate across the entire EEG data set. As can be seen from the two curves in the figure, the optimal segmentation point is 0.55. However, the sample size is not complete enough to demonstrate and fit an accurate ROC curve, so the value of 0.55 is not actually accurate and is only an approximate value. More EEG samples should be collected in subsequent studies to determine the accurate threshold. As the model accuracy of the default (0.5) of the model has been proved, the prediction results of the subsequent system design are still judged according to the default threshold of the model, but the specific probability value of the model here will be given as a reference. In addition, the value of curve AUC can reach 0.93 on the test set and 0.99 on the partial EEG data set. It can be seen that the output of this model is of great significance for the diagnosis of teachers' emotional stress relief in the process of Japanese teaching based on EEG analysis.

This paper established the recognition model of teachers' emotional stress relief in the process of Japanese teaching under the analysis of EEG signals and proved its superiority. The established model is the random forest model for classification using 12 features (calculated from signals of 10 EEG channels) mentioned above.

## 5. Conclusion

Both online and offline have their own characteristics, so they should be introduced into the evaluation method. However, if the two are separated, the overall teaching effect will be negatively affected. Promoting online and offline together in Japanese teaching evaluation system should be built in getting enough attention, the reason is that the online and offline two parts of teaching are not unrelated, but there is a connection relationship, such as EEG analysis under Japanese teaching process, the teacher mood is mainly convey knowledge and let students find difficult point, offline teaching is a difficult point for specific processing. If the teaching evaluation system with comprehensive guiding function cannot be constructed, the degree of connection between the two will be hindered. For example, in the evaluation of students' oral Japanese expression ability, teachers' emotions in the process of Japanese teaching based on EEG signal analysis can evaluate students' oral Japanese fluency. Offline teaching can allow students to have “real conversations” based on specific scenes, so as to evaluate students' coping ability. Teachers can combine the two evaluation results to find out the weaknesses of students and then make targeted responses. At present, deep learning and related computational memory, GPU and CPU are still in rapid development. We will continue to further optimize the deep learning model in this paper and further attempt to apply deep learning in EEG identification of teachers' emotions.

## Figures and Tables

**Figure 1:** Analysis and research on EEG signals of Japanese teachers' emotional stress elimination.

**Figure 2:** Experimental diagram of Japanese teachers' emotional stress elimination stimulus.

**Figure 3:** Flowchart of Japanese classroom teaching.

**Figure 4:** P-P diagram of average power spectral density based on positive and negative images.

**Figure 5:** ERSP results of the experimental group at F3 poles based on *t* test (*P* < 0.01).

**Figure 6:** ERSP results of normal group at F3 poles based on *T* test (*P* < 0.01).

**Figure 7:** ROC curve of the model.

**Table 1:** Main parameters of feature selection.

Method of feature selection	Parameters
Linear feature selection based on L1 (line feature)	Regularization parameter 0.03; (to select fewer features)
Feature selection based on tree model	The number of spanning trees is 3; the maximum depth is 4
FDR (false discovery rate) correction	FDR 0.03 (generally 0.05)

**Table 2:** How to regulate their own bad emotions?

Teacher answer	Number	Proportion
Sports, recreation	9	29%
Talk to family and friends	7	23%
Hope that through the understanding and help of others	6	16%
Negative ways like drinking, anger, etc.	5	15%
Ignore and sulk alone	5	9%
Analyze the causes of negative emotions, find out the root causes, and seek solutions	3	8%

**Table 3:** How do you regulate the negative emotions of the student group and individual?

Teacher answer	Number	Proportion
Infect your partner with your emotions	6	21%
Talk after class	16	62%
I do not really care	3	7%
Ignore and let students adjust themselves	4	10%

**Table 4:** Overall level of teachers' emotion management and descriptive analysis of each dimension.

Variable	*N*	Min	Max	Avg	Standard deviation	Mean standard deviation
Emotional awareness	388	6	25	15.89	3.78	3.89
Emotional expression	388	5	26	15.32	3.71	3.75
Emotional debugging	388	3	26	15.02	4.09	3.89
Emotional use	388	5	21	14.89	3.79	3.82
Emotional control	388	5	23	14.98	3.78	3.76
Emotional evaluation	388	5	18	14.32	3.23	3.67

**Table 5:** Statistical analysis of each pole between control group and normal group.

Pole	Ha	Sad	Pole	Ha	Sad
AF3	*P* < 0.05	*P* < 0.03	AF5	*P* < 0.02	*P* < 0.04
F7	*P* < 0.05	*P* < 0.01	F8	*P* < 0.01	*P* < 0.01
F7	*P* < 0.05	*P* < 0.05	F5	*P* < 0.04	*P* < 0.03
FC5	*P* < 0.05	*P* < 0.05	FC7	*P* < 0.05	*P* < 0.05
T7	*P* < 0.05	*P* < 0.01	T8	*P* < 0.01	*P* < 0.01
T7	*P* < 0.05	*P* < 0.05	T9	*P* < 0.05	*P* < 0.05

## Data Availability

The data used to support the findings of this study are included within the article.
